# Analysis of Transient Response of ZPW-2000A Jointless Track Circuit Considering Frequency Variation

**DOI:** 10.1155/2022/2257313

**Published:** 2022-04-30

**Authors:** Bin Zhao, Guanghao Yu, Dong Wang, Lei Chen, Jingning Ou

**Affiliations:** School of Automation & Electrical Engineering, Lanzhou Jiaotong University, Lanzhou 730070, China

## Abstract

In order to accurately analyze the influence of electromagnetic transient signals on the jointless track circuit when the electromagnetic transient signal propagates in the rail, it is necessary to consider the frequency-variable load terminated in the ZPW-2000A jointless track circuit and the frequency-variable loss inside the rail. A method is proposed for calculating the transient response of transmission lines system with frequency-variable end load of jointless track circuit. Firstly, the transmission lines model of jointless track circuit is established, based on multiconductor transmission lines theory, the model equation is deduced and discretized by finite difference time domain (FDTD). The vector fitting method is used to express the admittance of the tuning region in the track circuit, and the rational approximation function of the tuning region is derived from the poles, residues, and constants. The voltage and current at nodes in the tuning region are calculated by piecewise linear recursive convolution algorithm. Combined with the discrete transmission line equation, the current and voltage expression of the transient electromagnetic signal at the receiving end of the track circuit in time domain is obtained. Compared with state variable method, the error is less than 6%, which verifies the correctness of the proposed method. Finally, this paper studies the influence laws of different factors on the overvoltage at the receiving end of jointless track circuit and the weak links of jointless track circuit under the influence of transient electromagnetic signal. It provides theoretical reference for fault research and anti-interference analysis of ZPW-2000A jointless track circuit.

## 1. Introduction

Jointless track circuit is the key equipment used to detect the occupancy of train section, the integrity of rail, and the transmission of running information in railway line, which is an important basic equipment to ensure the safe operation of high-speed railway [1]. With the increasing complexity of railway construction environment, the rail and signal transmission equipment laid outdoors are easily disturbed by strong electromagnetic signals. Electromagnetic interference signals use rail as transmission medium to produce conduction interference or radiation coupled interference on jointless track circuits [2]. The investigations show that lightning strikes can cause failures of trackside tuning matching units, signal transmission cables and lightning protection analog network disks, transmitters and receivers, etc. Jointless track circuit is easy to make wrong responses by this disturbance, which will threaten the safety of train running. Therefore, it is important to analyze the interference of transient electromagnetic signal to track circuit.

The theory of multiconductor transmission lines is the theoretical basis of time-domain transient analysis of track circuits. Kunz and Luebbers [3] first solved the transmission lines equation by FDTD method, which provided a theoretical basis for time-domain solution of transmission lines. With the complex changes in transmission lines termination equipment, Wang et al. [4–6] respectively proposed a numerical algorithm based on Thevenin equivalent circuit method, state variable method, etc., to solve the terminal frequency-varying load and combined with the transmission line equation to solve the electromagnetic impulse response of the system. In the study of transient response of jointless track circuits. Mazloom et al. [7] proposed a method based on transmission line equation and ATP-EMTP simulation model to analyze the voltage response of track circuit at the moment of train entering and clearing. Zhao et al. [8] obtained the general solution of current and voltage of rail line by Laplace transformation of the transmission line equation of track circuit, which simplified the calculation model and ignored the electrical insulation section; Yong-jian [9] used the state variable method to analyze the receiving end of the DC track circuit and solved equation of the track circuit by combining the transmission line equation, but it was difficult to write the state equation when the circuit structure was complex. Zhichao et al. [10] analyzed the overvoltage of each signal equipment during lightning strike catenary by establishing lightning strike simulation model of signal system.

ZPW-2000A jointless rack circuit includes parallel nonlinear equipment and rail with frequency variation characteristics. In order to accurately calculate the electromagnetic transient response of track circuit transmission line system, the influence of terminating frequency variation load and rail frequency variation loss must be considered. Firstly, according to the transmission characteristics of ZPW-2000A jointless track circuit, the transmission line model of track circuit is established. The model cannot be calculated directly due to the presence of parallel or terminated nonlinear lumped elements in the track circuit. Based on the multiconductor transmission lines theory, the model equation is solved by FDTD. The vector fitting method is a powerful tool for the modeling analysis of frequency-dependent systems, which is used to fit the admittance of the tuning region. The rational approximation function of the track circuit is derived from the poles, residues, and constants. The relationship between voltage and current at both ends of the admittance is derived by piecewise linear recursive convolution, which is submitted into the discrete equation of transmission lines. Finally, the time-domain expression of the current and voltage at the receiving end of the track circuit is obtained. Compared with the state variable method, the error is less than 6%, which verifies the correctness of the proposed method. This method is used to analyze the influence of lightning stroke distance, electromagnetic signal frequency, and track bed resistance on the overvoltage at the receiving end of track circuit; it provides a theoretical basis for the anti-interference analysis of track circuit.

## 2. Modeling of Transmission Line of Track Circuit with Frequency-Variable Load Terminated

The outdoor equipment of jointless track circuit is composed of steel rail, tuning unit (BA), air-core coil (SVA), signal cable, matching unit and compensation capacitor, etc. The tuning unit and the air-core coil part form an electrical insulation section to prevent cross-zone signal transmission from adjacent sections. The compensation capacitor is used to improve the transmission performance of the track circuit and increase the transmission distance of the track circuit information. According to the transmission characteristics of track circuit, the rails are equivalent to uniform transmission lines [11]; it is characterized by two asymmetrical currents, one of which leaks into the ground, and the other flows from one rail to the other through ballast and sleepers. Taking a certain interval of track circuit as an example, the MTL equivalent model of jointless track circuit is established [12], as shown in Figure 1.

Here, *r*_1_ and *r*_2_ are the self-resistance of the rail; *l*_11_ and *l*_22_ are the self-inductance of the rail; *l*_12_ is the mutual inductance between rails; *g*_11_ and *g*_22_ are the leakage conductance between rails and Earth; *g*_12_ and *g*_21_ are the ballast resistance parameter of track characterized by conductance; *c*_11_ and *c*_22_ are the self-capacitance of the rail; *c*_12_ is the mutual capacity of the rails; and *z*_1_ and *z*_2_ represent the tuning region, respectively.

Transmission line losses are reflected in the conductor and the surrounding mediums; in general, these losses are frequency dependent, and the increase of frequency will lead to additional high-frequency losses. The most important is caused by the skin effect in the conductor and the polarization in the dielectric. Dielectric loss has little influence on transmission lines and can be ignored [12]. Therefore, the frequency domain expression of transmission line equation based on multiconductor transmission lines theory is

(1) $$\begin{array}{c} \frac{\text{d}\overset{⌢}{V}\left(z,w\right)}{\text{d}z}=\left[r\left(w\right)+jwl_{i}\left(w\right)\right]\hat{I}\left(z,w\right)-jwl\hat{I}\left(z,w\right)=-\hat{z}\left(w\right)\hat{I}\left(z,w\right), \end{array}$$

(2) $$\begin{array}{c} \frac{\text{d}\hat{I}\left(z,w\right)}{\text{d}z}=-g\left(w\right)\hat{V}\left(z,w\right)-jwc\hat{V}\left(z,w\right)=-\hat{y}\left(w\right)\hat{V}\left(z.w\right), \end{array}$$

where impedance and admittance are, respectively, $\hat{z}\left(w\right)={\hat{z}}_{i}\left(w\right)+jwl$, ${\overset{⌢}{z}}_{i}\left(w\right)=r\left(w\right)+jwl_{i}\left(w\right)$. $\hat{y}\left(w\right)=g\left(w\right)+jwc$.

Converting the frequency domain equations of (1) and (2) is transformed by Laplace transform into the time domain given the convolution equation as

(3) $$\begin{array}{c} \frac{\partial V\left(z,t\right)}{\partial z}=-z_{i}\left(t\right)*I\left(z,t\right)-l\frac{\partial I\left(z,t\right)}{\partial t}, \end{array}$$

(4) $$\begin{array}{c} \frac{\partial I\left(z,t\right)}{\partial z}=-gV\left(z,t\right)-c\frac{\partial V\left(z,t\right)}{\partial t}. \end{array}$$

In the case of high frequency, unit length resistance, internal inductance, and unit length conductance of conductor loss parameters are functions of frequency. The approximate formula $A+B\sqrt{\text{s}}$ for conductor losses is based on the transformation pair conversion; the inverse Laplace transform of the impedance in the conductor is

(5) $$\begin{array}{c} {\hat{z}}_{i}\left(s\right)=A+B\sqrt{s}=A+B\frac{1}{\sqrt{s}}s\Leftrightarrow A+B\frac{1}{\sqrt{\pi }}\frac{1}{\sqrt{t}}\frac{\partial }{\partial t}, \end{array}$$

where *A*=*r*_*dc*_, $B=r_{dc}/\sqrt{\pi }\sqrt{f_{0}}$, *r*_dc_ is DC resistance.

The convolution of the calculation in (3) is expressed as

(6) $$\begin{array}{c} z_{i}\left(t\right)*I\left(z,t\right)=\int_{0}^{t}z_{i}\left(\tau \right)I\left(z,t-\tau \right)\text{d}\tau \\ =AI\left(z,t\right)+B\frac{1}{\sqrt{\pi }}\int_{0}^{t}\frac{1}{\sqrt{\tau }}\frac{\partial I\left(z,t-\tau \right)}{\partial \left(t-\tau \right)}\text{d}\tau . \end{array}$$

The convolution term (6) is discrete with time step and divided by Δ*t* segment. Discrete convolution is approximated in the following way:

(7) $$\begin{array}{c} \int_{0}^{t}\frac{1}{\sqrt{\tau }}F\left(t-\tau \right)\text{d}\tau ≅\int_{0}^{\left(n+1\right)\Delta t}\frac{1}{\sqrt{\tau }}F\left(\left(n+1\right)\Delta t-\tau \right)\text{d}\tau \\ ≅\sum_{m=0}^{n}F^{n+1-m}\int_{m\Delta t}^{\left(m+1\right)\Delta t}\frac{1}{\sqrt{\tau }}\text{d}\tau =\sqrt{\Delta t}\sum_{m=0}^{n}F^{n+1-m}Z_{0}\left(m\right), \end{array}$$

where *F*(*t*)=∂*I*(*z*, *t*)/∂*t*, $Z_{0}\left(m\right)=\int_{m}^{m+1}1/\sqrt{\tau }\partial \tau$.

According to the FDTD algorithm, the position length of the transmission line is discretized by Δ*z*, and the time length is discretized by Δ*t*. The whole transmission lines are divided into *NDZ* segments, and the total solution times are divided into *NDT* segments. In order to ensure the stability of discrete calculation, the voltage of *NDZ* + 1 at discrete point *V*_1_, *V*_2_,…, *V*_*Z*_, *V*_NDZ+1_ and the discrete point current *I*_1_,*I*_2_,…, *I*_*NDT*_ does interleaving calculation. Then, (3), (4), and (7) can be discretized as

(8) $$\begin{array}{c} \frac{V_{k+1}^{n+1}-V_{k}^{n+1}}{\Delta z}+l\frac{I_{k}^{n+3/2}+I_{k}^{n+1/2}}{\Delta t}+A\frac{I_{k}^{n+3/2}+I_{k}^{n+1/2}}{2}+\frac{\sqrt{\Delta t}}{\sqrt{\pi }}B\sum_{m=0}^{n}\left[\frac{I_{k}^{n+3/2-m}+I_{k}^{n+1/2-m}}{\Delta t}\right]Z_{0}\left(m\right)=0,\\ \frac{I_{\text{k}}^{n+1/2}-I_{k-1}^{n+1/2}}{\Delta z}+g\frac{V_{k}^{n+1}+V_{k}^{n}}{2}+c\frac{V_{k}^{n+1}-V_{k}^{n}}{\Delta t}=0. \end{array}$$

The recursive relation of current at discrete points inside the transmission line is

(9) $$\begin{array}{c} I_{k}^{n+3/2}=F^{-1}\left(l\frac{\Delta z}{\Delta t}-A\frac{\Delta z}{2}+B\frac{1}{\sqrt{\pi }}\frac{\Delta z}{\sqrt{\Delta t}}Z_{0}\left(0\right)\right)I_{k}^{n+1/2}-F^{-1}B\frac{1}{\sqrt{\pi }}\frac{\Delta z}{\sqrt{\Delta t}}\sum_{m=1}^{n}\left[I_{k}^{n+3/2-m}-I_{k}^{n+1/2-m}\right],\\ Z_{0}\left(m\right)-F^{-1}\left(V_{k+1}^{n+1}-V_{k}^{n+1}\right),\\ F=l\frac{\Delta z}{\Delta t}+A\frac{\Delta z}{2}+B\frac{1}{\sqrt{\pi }}\frac{\Delta z}{\sqrt{\Delta t}}Z_{0}\left(0\right). \end{array}$$

## 3. Tuning Region Transient Modeling

In the ZPW-2000A jointless track circuit, the electrical insulation section realizes the electrical isolation of adjacent track and the stable output of local signal by forming series and parallel resonance for different carrier frequency signals. In the matching part, the rail impedance and cable impedance are matched to realize the output of high power signal to the rail [14]. The structure of electrical insulation section in jointless track circuit is shown in Figure 2.

Firstly, the transient model of tuning matching unit is established, and the drive point admittance of the tuning unit port is obtained by the short-circuit test method. The frequency domain admittance is fitted to a rational function expression by the vector matching method, as shown in (10). Secondly, the frequency domain rational function is transformed into time-domain expression by inverse Fourier transform. Finally, based on the piecewise linear recursive convolution method, the recursive iterative relation of admittance current is derived in (14). The admittance can be fitted to a rational function in the complex frequency domain by the vector matching method and the objective function *Y*(s) expresses its s-domain admittance in pole and residue form [13]:

(10) $$\begin{array}{c} Y\left(s\right)=\sum_{i=1}^{n}\frac{a_{i}}{s-c_{i}}+sh+g=\sum_{i=1}^{n}Y_{i}\left(s\right)+Y_{0}\left(s\right), \end{array}$$

where *n* is the order, *i* is an integer (*i* = 1,2,…, *n*); *a*_*i*_ is the residue, and *c*_*i*_ is the pole, both are real numbers or conjugate complex number pairs, sh is the coefficient of the first term, and *g* is the constant term.

The fitting order of the poles in the tuning area is 12 to achieve appropriate fitting effect. The amplitude characteristic and phase angle characteristic function are fitted according to the pole and residue values. Compared with the admittance model of the tuning unit, the results are shown in Figures 3 and 4.

The results of admittance fitting of the tuning element are consistent with those of the exact value and meet the requirements of calculation. According to the admittance rational function, the current equation of the connection node is derived. The voltage current relationship of the tuning unit in time domain is expressed as *I*_*z*_(*t*)=*Y*(*t*)*∗V*_*z*_(*t*). Defining two parameter variables [5],

(11) $$\begin{array}{c} \chi_{m}=\int_{m\Delta t}^{\left(m+1\right)\Delta t}Y\left(\tau \right)\text{d}\tau ,\\ \xi_{m}=\frac{1}{\Delta t}\int_{m\Delta t}^{\left(m+1\right)\Delta t}\left(\tau -m\Delta t\right)Y\left(\tau \right)\text{d}\tau . \end{array}$$

Using piecewise recursive convolution integral, we know that if the two variables are satisfied,

(12) $$\begin{array}{c} \rho =\frac{\xi_{m}}{\xi_{m-1}}=\frac{\chi_{m}}{\chi_{m-1}}. \end{array}$$

Then, the time-domain current *I*_*z*_^*n*^ can be written in the recursive iterative form:

(13) $$\begin{array}{c} I_{z}^{n+1}=\left(\chi_{0}-\xi_{0}\right)V_{z}^{n+1}+\xi_{0}V_{z}^{n}+\rho I_{z}^{n}. \end{array}$$

There are number of real numbers *N*_r_ and conjugate pairs *N*_g_ in the fitting residues of loads in residue regions and the poles, then the total current of the connected nodes is

(14) $$\begin{array}{c} I_{z}^{n+1/2}=PV_{z}^{n+1}+QV_{z}^{n}+I_{t}^{n+1}, \end{array}$$

where *P*=*χ*_0,*t*_ − *ξ*_0,*t*_+*g*/2+*h*/Δ*t*, *Q*=*χ*_0,*t*_+*g*/2 − *h*/Δ*t*;

(15) ξ0,t=12∑i=1Nrξ0,i+∑i=Nr+1Nr+NgReξ0,iχ0,t=12∑i=1Nrχ0,i+∑i=Nr+1Nr+NgReχ0,i,Itn=12∑i=1Nrρi+1Iz,in+∑i=Nr+1Nr+NgReρi+1Iz,in.

## 4. Transmission Line Voltage Equation of Track Circuit

When the transmission line load is pure resistance load, the current is *I*_0_=(*V*_0_ − *V*_1_)/*R*. The central difference method is used to discretize it.

(16) $$\begin{array}{c} I_{0}^{n+1/2}=\frac{\left(V_{0}^{n+1/2}-V_{1}^{n+1/2}\right)}{R}=\frac{1}{2R}\left[\left(V_{0}^{n+1}+V_{0}^{n}\right)\right.-\left.\left(V_{1}^{n+1}+V_{1}^{n}\right)\right]. \end{array}$$

According to the average value of power supply *I*_S_ current, (3) and (4) can be discretized:

(17) $$\begin{array}{c} \frac{1}{\Delta z/2}\left[I_{1}^{n+1/2}-\frac{I_{0}^{n+1}+I_{0}^{n}}{2}\right]+\frac{1}{2}g\left[V_{k}^{n+1}+V_{k}^{n}\right]+\frac{c}{\Delta t}\left[V_{k}^{n+1}-V_{k}^{n}\right]=0. \end{array}$$

The initial voltage expression of the transmission line equation of the track circuit is

(18) $$\begin{array}{c} V_{1}^{n+1}={\left(1+\frac{\Delta z}{\Delta t}cR_{s}+\frac{\Delta z}{2}gR_{s}\right)}^{-1}\left[\left(\frac{\Delta z}{\Delta t}Rc-\frac{\Delta z}{2}R_{s}g-1\right)V_{1}^{n}-2R_{s}I_{1}^{n+1/2}+2V_{0}^{n+1/2}\right]. \end{array}$$

The internal point voltage iteration formula of the equation is

(19) $$\begin{array}{c} V_{k}^{n+1}={\left(\frac{\Delta z}{\Delta t}c+\frac{\Delta z}{2}g\right)}^{-1}\left[\left(\frac{\Delta z}{\Delta t}c-\frac{\Delta z}{2}g\right)V_{k}^{n}-\left(I_{k}^{n+1/2}-I_{k-1}^{n+1/2}\right)\right]. \end{array}$$

According to the average value of load current *I*_L_ at the load at the end of the transmission line, the transmission line equation can be discretized as follows:

(20) $$\begin{array}{c} \frac{1}{\Delta z/2}\left[\frac{I_{L}^{n+1}+I_{L}^{n}}{2}\right.-\left.I_{\text{NDZ}}^{n+1/2}\right]+\frac{1}{2}g\left[V_{\text{NDZ}+1}^{n+1}+V_{\text{NDZ}+1}^{n}\right]+\frac{c}{\Delta t}\left[V_{\text{NDZ}+1}^{n+1}-V_{\text{NDZ}+1}^{n}\right]=0. \end{array}$$

When the nonlinear lumped element of a track circuit is terminated with a tuning unit as the terminal condition, the terminal condition gives the relation IL between voltage and current at the same time and position. According to (14), the current and voltage equation *I*_L_ at its endpoints is

(21) $$\begin{array}{c} I_{L}^{n+1/2}=P\left(V_{k+1}^{n+1}-V_{L}^{n+1}\right)+Q\left(V_{k+1}^{n}-V_{L}^{n}\right)+I_{t}^{n+1}. \end{array}$$

The terminal voltage equation of the transmission line equation of the track circuit is

(22) $$\begin{array}{c} V_{\text{NDZ}+1}^{n+1}={\left(P+\frac{c\Delta z}{2\Delta t}+\frac{g\Delta z}{4}\right)}^{-1}\left[\left(\frac{c\Delta z}{2\Delta t}-\frac{g\Delta z}{4}-Q\right)V_{\text{NDZ}+1}^{n}+PV_{L}^{n+1}+QV_{L}^{n}-I_{t}^{n}+I_{\text{NDZ}}^{n+1/2}\right]. \end{array}$$

## 5. Method Validation

To verify the validity of the constructed track circuit model and the transient response formula, taking P60 rail carrier frequency signal 2300 Hz and 1.4 km track section as an example, the lightning wave adopted the double exponential lightning electromagnetic signal with wave head of *T*_1_=1.2 *μ*s and wavelength of *T*_2_=50 *μ*s, recorded as 1.2/50 *µs* standard lightning wave [15], and the amplitude was 30 kA for simulation. According to the transmission line model of track circuit, the overvoltage of track surface at the receiving end of track circuit is solved. The state variable method is used to compare the response results with the proposed method.

It can be seen from Figures 5 and 6 that the numerical algorithm for transient response of track circuit proposed in this paper is consistent with the calculation results of state variable method. The calculation error is less than 6%.

### 5.1. Impact Tolerance Level of Signal Equipment

When the electromagnetic field induced by lightning reaches a certain level, the signal equipment will work improperly or be damaged. The lightning tolerance level of signal equipment terminals is obtained through the destructive lightning shock tolerance experiment, which is the key factor to determine the lightning resistance of signal system equipment [10], as shown in Table 1.

## 6. Analysis of Influencing Factors

### 6.1. Influence of Lightning Transmission Distance on Rail Surface Voltage

When lightning strikes the rail, the change of track surface overvoltage with distance between the lightning point and the tuning area of the track circuit is shown in Figure 7.

It can be seen from Figure 7 that with the increase of the distance between the lightning point and the receiving end of the track circuit, the rail surface overvoltage decreases rapidly with the increase of the distance. Especially when the transmission distance is less than 700 m, the overvoltage generated by lightning will exceed the withstand voltage range of the tuning unit end, and there is a risk of breakdown of trackside electronic equipment.

### 6.2. Considering the Influence of Different Frequencies on Rail Surface Voltage

In ZPW-2000A jointless track circuit, the rail is used as the transmission channel of frequency shift signal, and the rail parameters have the characteristics of frequency change. In the high-frequency electromagnetic environment, the load at the end of the transmission line usually shows the frequency change effect. In order to analyze the variation rules of signal overvoltage at the receiving end of track circuit when interference signals of different frequencies act on track circuit, the calculation results are shown in Figure 8.

In Figure 8, the simulation results show that the frequency of electromagnetic interference signal has a great influence on the voltage amplitude at the receiving end of the rail surface. At the same time, the higher the frequency of the interference signal is, the smaller the amplitude of the rail surface voltage is at the receiving end. With the increase of signal frequency, the rail impedance increases, the loss of interference signal on the track circuit increases, and the rail voltage amplitude decreases at the receiving end. The internal frequency loss of the transmission line is very little affected by the change of frequency and can be ignored in the future research.

### 6.3. Influence of Track Bed Resistance on Rail Surface Voltage

The primary side parameters of the jointless track circuit will affect the transmission of interference signals on the rail. The P60 rail is selected, its impedance value is a certain value, while the resistance of the track bed will change with the difference of ambient temperature and humidity [16]. In order to study the influence rule of track bed resistance on rail surface voltage at the receiving end of track circuit, when the resistance value of track bed is 2 Ω·km, 2.5 Ω·km, 4 Ω·km, and 5 Ω·km, the influence rule of different track bed resistance on rail surface overvoltage is analyzed, as shown in Figure 9.

As shown in Figure 8, the greater the ballast resistance is, the greater the overvoltage is. Meanwhile, the faster the rate of rise and attenuation of overvoltage are. With the decrease of track ballast resistance, the amplitude of rail surface voltage decreases at the receiving end.

## 7. Conclusion

1. The transient response model of track circuit is established. A numerical calculation method of transient electromagnetic response of track circuit transmission line system considering terminated frequency-varying load and frequency-varying loss is proposed, which is suitable for the analysis of transmission line model with terminated frequency-varying load. It provides theoretical reference for the transmission performance of jointless track circuits and the anti-interference design of track circuits.
2. The frequency of electromagnetic interference signal has great influence on the amplitude of rail voltage at the receiving end. However, the frequency has little effect on internal loss of rail. The overvoltage and the time of signal attenuation to stability increase with increasing of the ballast resistance.
3. According to withstand voltage level of the signal equipment, when the distance between the lightning strike point and the receiving end of the track circuit is small, there is a risk of insulation breakdown on the rail side of the tuning unit, so measures need to be taken to strengthen the protection of the signal equipment.

## Figures and Tables

**Figure 1:** Equivalent circuit diagram of track circuit transmission line.

**Figure 2:** Structural schematic diagram of tuning unit.

**Figure 3:** Vector fitting matches amplitude and model amplitude.

**Figure 4:** Vector fitting matches phase angle with model phase angle.

**Figure 5:** Comparison of calculation methods of overvoltage at receiving end of track circuit.

**Figure 6:** Error diagram of calculation results.

**Figure 7:** Influence of distance between lightning strike point and receiving end of track circuit on rail surface voltage.

**Figure 8:** Rail surface voltage at receiving end of track circuit with different frequencies.

**Figure 9:** Influence of ballast resistance on rail surface overvoltage.

**Table 1:** Lightning resistance of signal system.

Device	Port	Shock withstands voltage/kV
Power box	Power terminal	5 ∼ 8
Discrete component	(Resistance, capacitance) circuit	3 ∼ 5
Tuning matching unit	Rail side to cable side	15
Signal cable	Core pair shielding layer	10
	Core pair	15

## Data Availability

The data used to support the findings of this study are included within the article.
